RETRACTED

# The novel role of circular RNA ST3GAL6 on blocking gastric cancer malignant behaviours through autophagy regulated by the FOXP2/MET/mTOR axis

**DOI:** 10.1002/ctm2.707

**Published:** 2022-01-21

**Authors:** Penghui Xu, Xing Zhang, Jiacheng Cao, Jing Yang, Zetian Chen, Weizhi Wang, Sen Wang, Lu Zhang, Li Xie, Lang Fang, Yiwen Xia, Zhe Xuan, Jialun Lv, Hao Xu, Zekuan Xu

**Affiliations:** ^1^ Department of General Surgery the First Affiliated Hospital of Nanjing Medical University Nanjing China; ^2^ Collaborative Innovation Center for Cancer Personalized Medicine Nanjing Medical University Nanjing China; ^3^ Jiangsu Key Lab of Cancer Biomarkers, Prevention and Treatment, Collaborative Innovation Center for Personalized Cancer Medicine Nanjing Medical University Nanjing China

**Keywords:** autophagy, circST3GAL6, FOXP2, gastric cancer, transcription factor

## Abstract

Gastric cancer (GC) ranks third in mortality among all cancers worldwide. Circular RNAs (circRNAs) play an important role in the occurrence and development of gastric cancer. Forkhead box P2 (FOXP2), as a transcription factor, is closely associated with the development of many types of tumours. However, the regulatory network between FOXP2 and circRNAs remains to be explored. In our study, circST3GAL6 was significantly downregulated in GC and was associated with poor prognosis in GC patients. Overexpression of circST3GAL6 inhibited the malignant behaviours of GC cells, which was mediated by inducing apoptosis and autophagy. In addition, we demonstrated that circST3GAL6 regulated FOXP2 through the mir‐300 sponge. We further found that FOXP2 inhibited MET Proto‐Oncogene (MET), which was the initiating factor that regulated the classic AKT/mTOR pathway of autophagy. In conclusion, our results suggested that circST3GAL6 played a tumour suppressive role in gastric cancer through miR‐300/FOXP2 axis and regulated apoptosis and autophagy through FOXP2‐mediated transcriptional inhibition of the MET axis, which may become a potential target for GC therapy.

## Graphical abstract

This article revealed that the circST3GAL6 inhibits the proliferation and metastasis of gastirc cancer through autophagy regulated by circST3GAL6/miR‐300/FOXP2/MET/mTOR axis. Therefore, circST3GAL6 may serve as a prognostic marker and therapeutic target for gastric cancer.

## 1 INTRODUCTION

Gastric cancer (GC) is the third leading cause of death among all cancers worldwide. Based on the Global Cancer Statistics published in the American Journal of Clinical Oncology in 2018, GC ranks fifth in morbidity and third in mortality among all cancers. East Asia, including China, has a high incidence of gastric cancer.^1^, ^2^ Although much progress has been made in improving the quality of life of gastric cancer patients,^3^, ^4^, ^5^ the overall survival of GC patients was still not satisfactory in recent years.^6^ Hence, it is valuable to detect the potential mechanism and find possible clinical therapeutic targets.

RETRACTED

As noncoding RNAs, circular RNAs (circRNAs) are highly conserved and stable, which were formed in a closed circular loop without both 5′ caps and 3′ tails. CircRNAs have been detected in many organisms and have become a research hotspot in several years because of their unique stable structure.^7^, ^8^ Furthermore, circRNAs have been proved to have many significant effects in regulating translation, microRNA (miRNA) sponges and protein bindings.^9^, ^10^, ^11^ Increasing evidence has confirmed that circRNAs are involved in GC development by sponging miRNAs to regulate targeted genes.^12^ For example, circERBIN promotes the malignant behaviours of colorectal cancer (CRC) by miR‐125a‐5p sponges.^13^ Hence, we attempted to illustrate the mechanism of circST3GAL6 in gastric cancer.

As a transcription factor, the Forkhead box P (FOXP) family consists of FOXP1–4. FOXP proteins participate in regulating the transcription of genes associated with tumour progression.^14^ Although FOXP3 is a well‐known transcription factor, FOXP2 has rarely been investigated.^15^, ^16^ Recent studies have demonstrated that FOXP2 markedly affects cancer cell progression as a tumour suppressor.^17^ For example, FOXP2 suppressed the transcriptional activity of MET, and FOXP2 overexpression resulted in the transcriptional repression of MET.^18^ However, no related research has studied the association between circRNAs and FOXP2, and how FOXP2 is regulated by circRNAs remains to be solved.

Autophagy is essential to tumour progression, and circRNAs are reported to participate in cancer‐associated autophagy.^9^, ^19^ Additionally, the MET/mTOR axis regulates autophagy and promotes tumour metastasis.^20^

In the present study, we verified that circST3GAL6 is reduced in GC cells and tissues. Furthermore, we demonstrated that circST3GAL6 suppresses cell proliferation and metastasis by sponging miR‐300, affecting FOXP2 expression. CircST3GAL6 also regulates autophagy‐mediated proliferation and migration through the FOXP2/MET/mTOR axis. In conclusion, circST3GAL6 is expected to become a therapeutic target in the future.

1 **HIGHLIGHT**

- CircRNA ST3GAL6 promoted gastric cancer cell proliferation and metastasis in vitro and in vivo.
- CircST3GAL6 promoted gastric cancer progression through Forkhead box P2 (FOXP2)‐mediated autophagy by sponging miR‐300.
- CircST3GAL6 regulated the AKT/mTOR pathway through FOXP2 transcriptional inhibition of MET to regulate autophagy.

RETRACTED

## 2 MATERIALS AND METHODS

### 2.1 Cell lines and treatment

Human GC cell lines MGC‐803, BGC‐823, MKN‐45, SGC‐7901 and GES‐1 (normal stomach mucosa epithelium cells) were cultured in RPMI 1640 medium (Wisent, Shanghai, China) with 10% foetal bovine serum (FBS) (Wisent, Biocenter, China) and 1% penicillin‐streptomycin. While RPMI 1640 medium (Wisent) with 20% FBS (Wisent) was applied to culture HGC‐27 cells. All cells were cultured at 37°C in a humid atmosphere containing 5% CO_2_.

### 2.2 Tissue specimens/Tissue samples

All GC tissues in this study were gathered from GC patients undergoing radical gastrectomy in the Department of General Surgery of the First Affiliated Hospital of Nanjing Medical University. Samples were collected after surgical resection immediately and quickly frozen in liquid nitrogen. Histologic analyses were performed by a pathologist. TNM stage was determined according to the TNM Classification System (American Joint Committee on Cancer classification, 7th edition). Table 1 showed the clinical features of 60 GC patients.

**TABLE 1:** Expression of circST3GAL6 and miR‐300 in human gastric cancer and the clinicopathological characteristics of the patients’ *p < .05 and **p < .01 Statistically significant difference

		**circSTGAL6 expression**				**miR‐300 expression**			
**Parameters**	**Group**	**Cases**	**Low**	**High**	***p*‐value**	**Cases**	**Low**	**High**	***p*‐value**
Gender									
	Female	18	10	8	.5731	18	11	7	.2598
	Male	42	20	22		42	19	23	
Age at surgery									
	≥55	47	24	23	.754	47	22	25	.3472
	<55	13	6	7		13	8	5	
T grade									
	T1+T2	19	11	8	.5796	19	9	10	.999
	T3+T4	41	19	22		41	21	20	
Lymphatic invasion									
	Negative(N0)	8	2	6	.1287	8	3	5	.4475
	Positive(N1‐N3)	52	28	24		52	27	25	
Tumour site									
	Cardiac	24	10	14	.2918	24	11	13	.5982
	Non‐cardiac	36	20	16		36	19	17	
Stage									
	I–II	22	7	15	.0321^*^	22	13	9	.2839
	III–IV	38	23	15		38	17	21	
Size(cm)									
	<3	39	14	25	.0029^**^	39	24	15	.0149^*^
	≥3	21	16	5		21	6	15	
Lauren classification									
	Intestinal type carcinoma	21	13	8	.1760	21	9	12	.4168
	Diffuse gastric carcinoma	39	17	22		39	21	18	

*p* < 0.05 represents statistical significance (chi‐square test).

### 2.3 RNA‐seq analysis

TRIzol reagent (Invitrogen) was applied to collect RNA from GC tissues or cells. Next, PrimeScript RT Reagent (RR036A; TaKaRa, Japan) was used to reverse the transcription of the complementary DNA (cDNA). SYBR GREEN PCR Master Mix kit (4913914001; Roche, Shanghai, China) was used to a performed quantitative real‐time polymerase chain reaction (qRT‐PCR). Glyceraldehyde‐3‐phosphate dehydrogenase (GAPDH) and U6 were applied to normalize the messenger RNA (mRNA) and miRNA respectively. RiboBio (Guangzhou, China) provided all the specific primers for circRNAs. The sequencing statistics was attached in Table S3. Realgene (Nanjing, China) synthesized the PCR primer sequences of miRNAs and mRNAs. All the primers are presented in Table S1.

RETRACTED

### 2.4 Actinomycin D assay

5 × 10^4^ cells per well was suggested to inoculate in 24‐well plates and treated with 2 mg/L actinomycin D (MedChemExpress, China). The RNA was harvested at regular intervals (2, 4, 8 and 12 h). The expression of circST3GAL6 and ST3GAL6 mRNA were detected via qRT‐PCR.

### 2.5 Treatment of ribonuclease R

Note that, 3 U/mg of ribonuclease R (RNase R) was suggested to culture the RNA isolated from GC cells for 20 min at 37°C. The stable expression of circST3GAL6 and ST3GAL6 mRNA was detected via qRT‐PCR.

### 2.6 Plasmid construction and stable transfection

PcDNA3.1 vector (GenePharma, China) was the plasmid designed to contain cloned circST3GAL6 cDNA. Under the manufacturer's instruction, plasmids were transfected into cells.

### 2.7 Oligonucleotide transfection

Cells were seeded in 6‐well plates and incubated at 37°C in a humid atmosphere with 5% CO_2_ overnight. miRNA mimics, inhibitors and small interfering RNA (siRNAs) were designed and produced by GenePharma. Under the manufacturer's instruction, the above oligonucleotides were transfected into cells with lipofectamine 3000 (Thermo Fisher Scientific, USA).

### 2.8 Western blotting assay

RIPA buffer (P0013B; Beyotime Biotechnology, China) including phenylmethylsulfonyl fluoride were used to isolate protein from cells and tissues. A bicinchoninic acid method was applied to detect the protein concentration. The protein samples were resolved and separated by 8%–12% sodium dodecyl sulphate–polyacrylamide gel electrophoresis with an electrophoresis apparatus (Bio‐Rad, USA). After that, a polyvinylidene difluoride membrane was used to transfer proteins. Then the membrane was blocked by incubating with Quick Block (P0252; Beyotime Biotechnology) for 20 min. Next, the membranes were treated with a primary antibody, using GAPDH as an internal reference at 4°C overnight. At last, a corresponding secondary antibody was applied to steep the membranes at room temperature for 2 h. Enhanced chemiluminescence detection was used to detect the protein on the blots.

### 2.9 Cell counting kit‐8 assay

Treated cells were inoculated at 10^4^ cells per well in 96‐well plates and then mixed 10 μl of cell counting kit‐8 (CCK‐8) solution (Dojindo Laboratories, Japan) with 90 ul medium to each well every other day. After culturing for 2 h at 37°C, we recorded the absorbance of the cells at 450 nm with a microplate reader (BioTek, USA).

RETRACTED

### 2.10 Colony formation assay

GC cells were inoculated in different 6‐well plates. Each well was inoculated with 10^3^ cells, and then the 6‐well plates were cultured for 2 weeks in an incubator containing 5% CO2. Two weeks later, the cell proliferation state was observed after staining the cells.

### 2.11 5‐Ethynyl‐2′‐deoxyuridine assay

We inoculated the transfected cells in 96‐well plates at 10^4^ per well and cultured them for 24 h. The next day, 5‐ethynyl‐2′‐deoxyuridine (EdU) solution (RiboBio) was added to each well of the 96‐well plate for incubation. After that, the cells were fixed and then were subjected to Apollo staining and DNA staining using Apollo reaction solution and Hoechst 33342, respectively. Finally, we observed the red and blue signals under the microscope to evaluate cell proliferation.

### 2.12 Transwell assay

First, we added 600 μl of complete medium to the lower side of the Transwell chambers. Next, we diluted the cells with serum‐free RMPI‐1640 medium to 2 × 10^4^/ml and then added 200 ul medium to the upper layer of Transwell chambers (Millipore, USA). After incubation for 24 h in an incubator containing 5% CO_2_, we fixed and stained the cells with 75% alcohol and crystal violet respectively. Finally, we cleaned chambers with PBS and then used cotton swabs to remove the cells that did not penetrate the chamber.

### 2.13 Flow cytometric analysis

First, we seeded the transfected cells in 6‐well plates. Next, we collected all the cells and incubated them using the Apoptosis Detection Kit reagents (BD Pharmingen, USA) for 2 days. After 15 min of incubation, we observed the cells using CELL Quest software (BD Biosciences, USA). The percentage of apoptosis cells is reflected by the corresponding quadrant on the apoptosis map.

### 2.14 Fluorescent in situ hybridization

First, paraformaldehyde was applied to immobilize cells for 15 min. Then, cells were incubated overnight in 70% ethanol at 4°C. Next, cells were infiltrated with 0.5% Triton X‐100 for 5 min and then cleaned with saline sodium citrate buffer. Then, the cells were hybridized with a labelled circRNA or miRNA fluorescent in situ hybridization (FISH) probe in a hybridization buffer at 37°C overnight. At last, the nucleus was stained with 4,6‐diamidino‐2‐phenylindole (DAPI) for 5–10 min. At last, we captured the images by a fluorescence microscope.

### 2.15 Pull‐down assay

A biotin‐labelled probe for circST3GAL6 was designed by RiboBio. The cells were harvested and then incubated overnight with circST3GAL6 probes or control oligonucleotide probes at 4°C. The mixture of RNA and probes were combined with the magnetic bead several times using a washing buffer. After that, the RNA was collected via a specific RNA extraction kit (QIAGEN, Germany) and detected by qRT‐PCR. Biotinylated miR‐300 probes and miR‐NC probes were manufactured by GenePharma.

RETRACTED

### 2.16 Immunohistochemical analysis of tissue samples

The GC tissues or subcutaneous tumours were immobilized with 10% formalin and then placed in paraffin. Next, the tissues were sliced into slides and incubated with the corresponding primary antibody overnight at 4°C. The slices were then incubated with the secondary antibody (ABCAM, UK) of the corresponding species for 1 h at 37°C. At last, slices were observed via an optical microscope. Immunohistochemical (IHC) score = Frequency*intensity. The frequency is classified by the proportion of positive cells. The classification is as follows: grade 0, grade 1, grade 2, grade 3 and grade 4; the proportion of positive cells represents <5%, 5%–25%, 25%–50%, 50%–75% and more than 75%, respectively. The cell intensity staining is classified as 0, 1, 2 and 3, which means negative, weak, moderate and strong, respectively.

### 2.17 Transmission electron microscope

Note that, 2.5% glutaraldehyde was used to fix the cell deposits at 4°C overnight. Then the samples were removed and fixed in 1% osmium tetroxide for 60 min at room temperature. Next, the samples were encased in 10% gelatin and then dehydrated for 10 min in increasing alcohol concentrations (30%, 50%, 70%, 90%, 95% and 100% × 3). Next, the epoxy propane was permeated with increasing concentrations (25%, 50%, 75% and 100%). The sample was then placed in a pure Quetol‐812 epoxy resin and polymerized for 12 h at 35°C, 12 h at 45°C and 24 h at 60°C. Finally, the samples were cut into slices (100 nm), using an ultrathin slicer, which were then stained with uranyl acetate and lead citrate for 10 min and 5 min, separately. At last, we observed the sections under a transmission electron microscope (TEM) of 120 kV.

### 2.18 Nude mouse xenograft model

In total, 1 × 10^6^ treated GC cells suspended in PBS were injected into the groin of 5‐week‐old nude mice, which were purchased from the Department of Laboratory Animal Center of Nanjing Medical University. After 4 weeks, all mice were sacrificed and tumours were isolated to measure their weight and volume. The tumour volume was calculated as V = length × width^2^ × 1/2.

### 2.19 In vivo metastasis assay

1 × 10^6^ stably transfected GC cells were injected into 5‐week‐old nude mice by tail vein injection. The bioluminescent signals of lung metastasis were observed using a specific imaging system (Caliper Life Sciences, USA) after 4–5 weeks. The lung metastatic lesions were assessed via haematoxylin and eosin‐stained sections.

RETRACTED

### 2.20 Luciferase reporter assay

Cells were seeded in 24‐well plates and co‐transfected with the miRNA mimics and plasmids. The luciferase signals after transfection for 48 h were detected via a luciferase reporter assay instrument (Promega, Madison, WI). Renilla luciferase activity was used to normalize the detected luciferase activity.

### 2.21 Confocal microscopy

Cells were transfected with Green Fluorescent Protein‐Red Fluorescent Protein‐LC3 lentivirus (GeneChem, China) and inoculated into specific small Petri dishes for confocal microscopy. The nuclei were stained with DAPI. Confocal microscopy (Carl Zeiss, Germany) was applied to detect the different signals. Red spots represent autolysosomes while yellow spots represent autophagosomes. Three random fields were selected for puncta quantification.

### 2.22 Chromatin immunoprecipitation assay

Chromatin immunoprecipitation (ChIP) assays were conducted with the Magna ChIP A/G Chromatin Immunoprecipitation Kit (17–10085; Millipore Sigma, USA) under the manufacturer's protocol. Cells were fixed with 37% formaldehyde. The chromatin was fragmented by ultrasonic fragmentation on ice and immunoprecipitation was performed with normal immunoglobulin G and FOXP2 antibodies (5337; Cell signalling technology). The products were washed with washing buffer and DNA was purified to remove the protein and obtain the purified DNA product. Finally, PCR was used to detect the results.

### 2.23 Statistics

In each experiment, data were expressed as mean ± SD. *p* < .05 was determined as a significant difference. Student's *t*‐test and one‐way analysis of variance were performed.

## 3 RESULTS

### 3.1 CircST3GAL6 expression profiles in gastric cancer

To screen circRNAs participated in the progression of gastric cancer, the circRNA‐seq assay was applied to analyse different expression profiles of circRNAs in three paired GC tissues and normal stomach tissues. Finally, 121 differentially expressed circRNAs were obtained, of which 76 were upregulated and 45 were downregulated (log_2_FoldChange ≥2 or ≤0.5, *p* < .05). Next, we excluded circRNAs that were not included in circbase^21^ and obtained 90 circRNAs. We chose the top 20 circRNAs to generate a heat map according to the log_2_Foldchange (Figure 1A). Circ_0066608, which is also called circST3GAL6, attracted our attention because of its most significant low expression in GC (Figure 1B). We collected a cohort of 60 paired GC tissues and normal stomach tissues to verify circST3GAL6 expression. Among them, circST3GAL6 was significantly downregulated via qRT‐PCR (Figure 1C). Additionally, the overall survival of GC patients with lower expression of circST3GAL6 was worse according to the overall survival analysis of circST3GAL6 expression in 60 GC patients (Figure 1D). Furthermore, the level of circST3GAL6 detected in the gastric cancer cell lines was lower than that in the GES‐1 cell line. Among them, the expression of circST3GAL6 in the BGC‐823 cell line was the lowest, followed by the SGC‐7901 cell line (Figure 1E). Therefore, the BGC‐823 and SGC‐7901 GC cell lines were selected to study the potential mechanism of circST3GAL6 affecting GC. Additionally, we observed that circST3GAL6 expression was negatively correlated with tumour stage and size by analysing the clinical data of the above 60 patients (Table 1). In summary, circST3GAL6 is significantly reduced in GC cells tissues, which deserves further study.

RETRACTED

**FIGURE 1:** CircST3GAL6 expression profiles in gastric cancer tissues and paired normal gastric tissues and identification of the structure and characteristics of circST3GAL6. (A) A cluster heat map was used to show the expression variations of these top 20 circRNAs transcripts in tumour tissues relative to matched normal tissues. (B) Volcano map showed the differences in the expression of circRNAs in gastric cancer (GC) tissues and adjacent normal tissues. (C) Quantitative real‐time polymerase chain reaction (qRT‐PCR) showed that the expression of circST3GAL6 in GC tissues was significantly lower than that in adjacent normal tissues. (D) Overall survival analysis based on circST3GAL6 expression in 60 GC patients. (E) Different expression levels of circST3GAL6 in GC cell lines. (F) Confirmation of head‐to‐tail splicing of circST3GAL6 with Sanger sequencing. (G) CircST3GAL6 and ST3GAL6 mRNA were treated with RNase R to detect their stability via qRT‐PCT. (H) qRT‐PCR analysis of circST3GAL6 and ST3GAL6 after actinomycin D treatment. (I) qRT‐PCR products of linear and circular products amplified with convergent and divergent primers in cDNA and genomic DNA (gDNA) compared to Glyceraldehyde‐3‐phosphate dehydrogenase (GAPDH). (J) FISH experiments showed that CircST3GAL6 was mostly located in the cytoplasm. (K) The proportion of circST3GAL6 in the nucleus and cytoplasm was confirmed by qRT‐PCR. (*p < .05, **p < .01, ***p < .001. Data are expressed as the means ± SDs)

### 3.2 Identification of the structure and characteristics of circST3GAL6

It was found that circST3GAL6 was located on chromosome 3 and formed a loop by connecting head to end with exon 2–5, as confirmed by Sanger sequencing. Next, primers were designed to perform qRT‐PCR and we found that circST3GAL6 could resist digestion by RNase R treatment, but not linear ST3GAL6 or GAPDH (Figure 1G). Furthermore, it was shown that circST3GAL6 was more resistant to actinomycin D degradation than linear ST3GAL6 (Figure 1H). Additionally, agarose gel electrophoresis was applied to investigate the expression of ST3GAL6 and GAPDH in gDNA and cDNA of GC cells respectively. We checked circST3GAL6 expression in cDNA with different primers and found that circST3GAL6 could not be amplified in gDNA products by divergent primers, which confirmed that circST3GAL6 was not generated by genomic rearrangement (Figure 1I). FISH assay and qRT‐PCR analysis of cytoplasmic and nuclear RNA proved that circST3GAL6 was predominantly located in the cytoplasm (Figure 1J,K). Thus, the above results indicated that circST3GAL6 is a real circRNA mostly located in the cytoplasm.

RETRACTED

### 3.3 CircST3GAL6 inhibits malignant behaviour and promotes apoptosis and autophagy in vitro

To verify whether circST3GAL6 affects the malignant behaviour of GC cells, specific siRNAs were designed to silence circST3GAL6 expression and constructed a circST3GAL6 overexpression plasmid. The transfection efficiency of circST3GAL6 was verified via qRT‐PCR, while ST3GAL6 mRNA was not affected (Figure S1A,B). Next, we performed functional experiments to verify the functions of circST3GAL6 on the biological behaviour of GC cells. We demonstrated that circST3GAL6 overexpression significantly inhibited the proliferation rate of GC cells (Figure 2A–C and Figure S1C,D) and promoted cell apoptosis (Figure 2E and Figure S1H), as indicated by CCK‐8, colony formation, EdU, and Annexin V‐FITC apoptosis detection assays. Additionally, knockdown of circST3GAL6 promoted cell proliferation (Figure 2A–C and Figure S1C,D) and inhibited cell apoptosis (Figure 2E and Figure S1H). The above results indicated that circST3GAL6 expression was significantly negatively correlated with GC cell growth. In order to confirm the connection between circST3GAL6 and cell apoptosis, the relevant apoptosis proteins were detected via western blotting. CircST3GAL6 overexpression significantly increased the protein level of cleaved Caspase‐3, while Bcl‐2 was downregulated and circST3GAL6 knocking down showed the opposite results, which are shown in Figure 2G and Figure S1J,K. Since apoptosis has been reported to affect the level of autophagy,^22^, ^23^ we tried to discover whether circST3GAL6 affects autophagy. GFP/mRFP‐LC3 dot accumulation was observed by overexpressing circST3GAL6, while circST3GAL6 knockdown showed opposite results (Figure 2F and Figure S1I). Next, we detected p62 and LC3 I/II levels in GC cells by western blotting, and circST3GAL6 overexpression raised the rate of LC3 II/I and reduced expression of p62 (Figure 2G and Figure S1J,K). Additionally, we found that circST3GAL6 overexpression reduced the metastatic ability of GC cells, while circST3GAL6 knockdown showed opposite results (Figure 2D and Figure S1E–G) via Transwell assays, showing that circST3GAL6 was negatively correlated with GC cell metastasis. Because the epithelial‐mesenchymal transition (EMT) is related to metastasis of cancer cells,^24^ we investigated the role of circST3GAL6 in regulating EMT‐related factors. We observed downregulated N‐cadherin, vimentin, slug, snail and upregulated expression of E‐cadherin in cells transfected with circST3GAL6 overexpression plasmids. Meanwhile, GC cells transfected with siRNA displayed the opposite results. (Figure 2G and Figure S1J,K). In summary, the above results verify that circST3GAL6 plays a key role in inhibiting the proliferation, metastasis of GC cells.

RETRACTED

**FIGURE 2:** CircST3GAL6 inhibits the proliferation, metastasis and promotes apoptosis, autophagy of gastric cancer (GC) cells in vitro. (A) The proliferation of BGC‐823 and SGC‐7901 cells transfected with circST3GAL6 siRNA or an overexpression plasmid by a CCK‐8 assay. (B) The effect of circST3GAL6 on was cell proliferation examined by colony formation assay in BGC‐823 and SGC‐7901 cells. (C) The effect of circST3GAL6 on was cell proliferation examined by 5‐ethynyl‐2′‐deoxyuridine (EdU) assay in BGC‐823 and SGC‐7901 cells, scale bar = 100μm. (D) The effect of circST3GAL6 on cell migration was evaluated by Transwell assay. (E) The effect of circST3GAL6 on modulating cell apoptosis was evaluated by flow cytometry assay. (F) The effect of circST3GAL6 on GFP/mRFP‐LC3 dots in BGC‐823 and SGC‐7901 cells were observed and counted by confocal microscopy, scale bar = 20μm. (G) Detection of apoptosis, autophagy and epithelial‐mesenchymal transition (EMT) related proteins by western blotting in BGC‐823 and SGC‐7901 cells. (*p < .05, **p < .01, ***p < .001. Data are expressed as the means ± SDs)

### 3.4 CircST3GAL6 inhibits tumour growth and metastasis in vivo

We injected 1 × 10^6^ GC cells into nude mice transfected with circST3GAL6 overexpression or sh‐circST3GAL6 subcutaneously to verify the effect of circST3GAL6 in vivo. The mice of three groups were sacrificed after 4 weeks, and tumours were measured respectively (Figure 3A). Results from the negative control group were used as a baseline, the tumour weight and volume of the circST3GAL6 overexpression group were significantly reduced, while sh‐circST3GAL6 showed the opposite results (Figure 3B). Next, the tumour tissues were made into slices and immunohistochemically stained with Ki‐67. Lower expression of Ki‐67 was observed in the circST3GAL6 overexpression group while the circST3GAL6 knocking down group showed the stronger Ki‐67 staining (Figure 3C). Furthermore, we established a model of lung metastasis. After GC cells were injected into the tail veins of nude mice, we observed the luciferase signals 4 weeks later. CircST3GAL6 overexpression significantly inhibited metastasis to the lung, while circST3GAL6 knockdown promoted lung metastasis (Figure 3D). The lung tissues of mice were separated, and haematoxylin‐eosin staining was applied to detect the formation of lung metastases, results of which were consistent with the luciferase signals (Figure 3E). In conclusion, the above results proved that circST3GAL6 inhibits tumour proliferation and metastasis in vivo.

RETRACTED

**FIGURE 3:** CircST3GAL6 inhibits tumour growth and metastasis in vivo. (A) Overexpression of circST3GAL6 inhibited the growth of xenograft tumours, while knockdown of circST3GAL6 promoted tumour growth. (B) The volume and weight of xenograft tumours were measured. (C) The tumour tissues were stained with Ki67 antibody, scale bar = 20 μm. (D) Overexpression of circST3GAL6 inhibited lung metastasis, while knockdown of circST3GAL6 promoted lung metastasis and the relative level of radiancece were measuresd (E) Hematoxylin‐eosin staining showed the size of lung metastatic tissues and the number of lung metastatic lesions were measured; scale bar = 200 μm. (*p < .05, **p < .01, ***p < .001. Data are expressed as the means ± SDs)

### 3.5 CircST3GAL6 functions as a miRNA sponge of miR‐300

CircRNAs have been reported to sponge miRNAs and regulate downstream genes in tumour development.^25^, ^26^ Target miRNAs of circST3GAL6 were predicted using two prediction databases: miRanda^27^ and PITA.^28^ According to the intersection of these two databases, seven miRNAs (hsa‐miR‐300, hsa‐miR‐370‐5p, hsa‐miR‐510‐5p, hsa‐miR‐6758‐5p, hsa‐miR‐6832‐5p, hsa‐miR‐6859‐5p and hsa‐miR‐877‐5p) were selected based on binding scores (Figure 4A). To absorb circST3GAL6‐related miRNAs, we performed pull‐down assays using a specific biotin‐labelled circST3GAL6. The efficiency of the circST3GAL6 probe is shown in Figure 4B. qRT‐PCR was applied to detect the expressions of these miRNAs in the pull‐down assay. Among these miRNAs, only miR‐300 was found to be significantly enriched with circST3GAL6 in both cells, while the rest of miRNAs did not interact so closely with circST3GAL6 (Figure 4C). Additionally, two binding sites between miR‐300 and circST3GAL6 were forecasted and confirmed via the luciferase reporter assay (Figure 4D). When we cotransfected wild‐circST3GAL6 and miR‐300, we observed reduced luciferase reporter activity compared with cotransfection with control RNA. Next, we mutated two binding sites in the circST3GAL6 sequence and found that the cotransfection of miR‐300 and mut‐circST3GAL6, with both binding sites mutated, did not significantly reduce the luciferase signal (Figure 4E). In conclusion, the direct connection between circST3GAL6 and miR‐300 was proved. Moreover, we performed FISH assays and found that miR‐300 and circST3GAL6 were co‐located in the cytoplasm (Figure 4F). MiR‐300 expression was significantly upregulated on 60 paired GC tissues and adjacent normal stomach tissues via qRT‐PCR (Figure 4G). Meanwhile, the negative correlation between circST3GAL6 and miR‐300 was confirmed (Figure 4H). According to the clinical features of the above patients, miR‐300 was related to GC tumour size, which is shown in Table 1. Furthermore, we performed the FISH assay in 15 paired GC and adjacent tissues to detect the relation between miR‐300 and circST3GAL6 (Figure 4I), which showed similar trends with the former results.

RETRACTED

**FIGURE 4:** CircST3GAL6 functions as a microRNA (miRNA) sponge of miR‐300. (A) Venn diagram showing the target miRNAs of circST3GAL6 predicted by miRanda and PITA. (B) The expression of circST3GAL6 in BGC823 and SGC7901 cell lysates was detected via quantitative real‐time polymerase chain reaction (qRT‐PCR). (C) qRT‐PCR analysis to examine the expression of candidate miRNAs after pull‐down assays in BGC‐823 and SGC‐7901 cells. (D) Sequence diagram of the binding sites between circST3GAL6 and miR‐300. (E) Analysis of luciferase activity in BGC823 and SGC7901 cells transfected with WT or MUT miR‐300. (F) FISH assay showed that circST3GAL6 and miR‐300 were co‐localized in the cytoplasm of BGC‐823 and SGC‐7901 cells. Scale bar = 100 μm. (G) qRT‐PCR showed that the expression of miR‐300 in gastric cancer (GC) tissues was significantly higher than that in adjacent normal tissues. (H) qRT‐PCR showed that the levels of circST3GAL6 and miR‐300 were negatively correlated. (I) FISH assay of circST3GAL6 and miR‐300 in 15 paired GC and adjacent tissues from patients. FISH scores were measured. Scale bar = 50 μm. (*p < .05, **p < .01, ***p < .001. Data are expressed as the means ± SDs)

As the above results proved that circST3GAL6 could sponge miR‐300, we attempted to find out whether the tumour suppressor role of circST3GAL6 was miR‐300 dependent. Then we constructed the circST3GAL6 mutant plasmid which blocked the connection between circST3GAL6 and miR‐300 (Figure S3A). The functional experiments showed that circST3GAL6 MUT could restore the effect of circST3GAL6 wild type on cell proliferation, apoptosis and metastasis (Figure S3B–D). Furthermore, confocal microscopy was applied to detect the level of autophagy. CircST3GAL6 MUT could significantly restore the effect of circST3GAL6 on GFP/mRFP‐LC3 dots (Figure S3F). Finally, the protein level of apoptosis, autophagy and EMT related proteins were detected and showed the same results with the functional experiments (Figure S3G). To sum up, these results proved that the effect of circST3GAL6 is miR‐300 dependent.

RETRACTED

### 3.6 MiR‐300 overexpression could restore the functions of circST3GAL6 on GC cells

To verify whether circST3GAL6 affected malignant biological behaviour in GC cells via the circST3GAL6/miR‐300 axis, we performed rescue experiments. First, we detected the transfection efficiency of miR‐300 inhibitors and mimics (Figure S2A,B). MiR‐300 overexpression promoted the proliferation and metastasis of GC cells and inhibited GC cell apoptosis, which was verified by Transwell assays, colony formation assay, EdU assay, and Annexin V‐FITC apoptosis detection assays (Figure 5A–E and Figure S2C–E). Furthermore, miR‐300 mimics restored the negative effects of circST3GAL6 overexpression on proliferation, metastasis, as well as apoptosis (Figure 5A–E and Figure S2C–E). Apoptosis‐ and EMT‐related protein expression were subsequently detected through western blotting assay. The effect of circST3GAL6 overexpression on cleaved Caspase‐3, Bcl‐2 and EMT‐related protein levels was restored by miR‐300 mimics (Figure 5J,K and Figure S2H,I). Since circST3GAL6 has been confirmed to be related to autophagy, we further explored the function of miR‐300 on autophagy. Interestingly, miR‐300 mimics could reverse the increase in the signals of GFP/mRFP‐LC3 caused by circST3GAL6 overexpression (Figure 5H,I and Figure S2F,G). Increased rate of LC3 II/I and downregulated p62 protein level caused by circST3GAL6 overexpression were reversed by miR‐300 mimics (Figure 5J,K and Figure S2H,I). Furthermore, miR‐300 mimics could restore the effect of circST3GAL6 overexpression on tumour growth (Figure S4A,B). These results demonstrated that circST3GAL6 could play a tumour‐suppressive role and regulate autophagy by sponging miR‐300.

**FIGURE 5:** Overexpression of miR‐300 reverses the effect of circST3GAL6 on gastric cancer (GC) cells. (A,B) miR‐300 mimics could restore the effect of circST3GAL6 on cell proliferation in BGC‐823 and SGC‐7901 cells by colony formation assays. (C,D) miR‐300 mimics could restore the effect of circST3GAL6 on cell proliferation in BGC‐823 and SGC‐7901 cells by EDU assays, scale bar = 100μm. (E) The promotion of cell apoptosis by circST3GAL6 overexpression was restored by miR‐300 mimics in BGC‐823 and SGC‐7901 cells. (F,G) The inhibition of cell migration and invasion by circST3GAL6 overexpression was restored by miR‐300 mimics in BGC‐823 and SGC‐7901 cells. (H,I) The effect of circST3GAL6 overexpression on autophagy can be recovered by miR‐300 in BGC‐823 and SGC‐7901 cells, scale bar = 20μm. (J) Expression levels of apoptotic, epithelial‐mesenchymal transition (EMT) and autophagy proteins were examined by western blotting in BGC‐823 and SGC‐7901 cells. (*p < .05, **p < .01, ***p < .001. Data are expressed as the means ± SDs)

RETRACTED

### 3.7 FOXP2 is a target of circST3GAL6 by sponging miR‐300

Based on the results above, we further studied the downstream mechanism of miR‐300. We employed miRWalk,^29^ miRDB^30^ and TargetScan^31^ and combined with the significantly downregulated genes in The Cancer Genome Atlas (TCGA) GC database. Ten genes overlapped (Figure 6A) and qRT‐PCR demonstrated that FOXP2 was significantly upregulated in both GC cells after transfecting with miR‐300 inhibitors, illustrating that FOXP2 may become the potential binding target of miR‐300 in GC (Figure 6B). The bioinformatics tool TargetScan was applied to predict the binding base sequence between miR‐300 and the 3′UTR of FOXP2 (Figure 6C). As shown in Figure 6D, we found that miR‐300 overexpression could decrease the luciferase signal of wild‐type FOXP2 rather than mutant FOXP2 in GC cells, indicating that miR‐300 could connect to the 3′UTR of FOXP2. TCGA database revealed that FOXP2 was significantly reduced in GC tissues (Figure 6E). Furthermore, it was shown that FOXP2 expression was lower in 60 paired GC tumour tissues than that in normal tissues via qRT‐PCR (Figure 6F). Besides, the expression of circST3GAL6 and FOXP2 was positively correlated. (Figure 6G). Subsequently, circST3GAL6 overexpression upregulated the expression level of FOXP2, which could be inhibited by miR‐300 mimics via qRT‐PCR and western blotting assay (Figure 6H and Figure S5A). Finally, IHC analysis of 12 paired GC tumour tissues confirmed that the degree of FOXP2 staining in gastric cancer tissues was lower than that in normal gastric tissues (Figure 6I). On the basis of the above results, we proved the potential regulation of FOXP2 by circST3GAL6 through sponging miR‐300.

**FIGURE 6:** Forkhead box P2 (FOXP2) is a target of circST3GAL6 by sponging miR‐300. (A) Venn diagram of target genes of miR‐300 predicted by miRWalk, miRDB, Targetscan and down‐regulated genes of The Cancer Genome Atlas (TCGA). (B) Quantitative real‐time polymerase chain reaction (qRT‐PCR) analysis of the relative levels of the 10 candidate genes in BGC‐823 and SGC‐7901 cells transfected with miR‐300 inhibitor or negative control. (C) Schematic of potential binding site of miR‐300 for FOXP2. (D) Luciferase reporter assay for determining whether miR‐300 could bind to wt‐FOXP2–3′UTR or mut‐FOXP2–3′UTR. (E) The TCGA database showed that the expression of FOXP2 in gastric cancer (GC) tissues was significantly lower than that in normal tissues. (F) qRT‐PCR showed that FOXP2 was significantly lower in GC tissues. (G) qRT‐PCR showed that the expression levels of circST3GAL6 and FOXP2 were positively correlated. (H) Overexpression of miR‐300 could restore the effect of CircST3GAL6 on FOXP2 expression by qRT‐PCR and western blotting in BGC‐823 cell. (I) Immunohistochemistry showed that the expression of FOXP2 was lower in GC tissues than that in adjacent normal tissues; scale bar = 200 μm. (*p < .05, **p < .01, ***p < .001. Data are expressed as the means ± SDs)

RETRACTED

### 3.8 Knockdown of FOXP2 reverses the functions of miR‐300 inhibitors on GC cells

Because we have proved that circST3GAL6 played a tumour‐suppressor role by sponging miR‐300 and FOXP2 was the downstream gene of miR‐300, we tried to find out how circST3GAL6 regulates FOXP2 via miR‐300 and its effects on GC cells. The transfection efficiency of FOXP2 siRNAs and overexpression plasmids was verified (Figure S5B). The promotion of proliferation of GC cells caused by miR‐300 knockdown could be restored via FOXP2 knockdown (Figure 7A–D). Transfection with miR‐300 inhibitors promoted GC cell apoptosis, and FOXP2 knockdown restored this effect (Figure 7E). The functions of miR‐300 inhibitors on metastasis could also be restored by FOXP2 knockdown (Figure 7F,G). The protein level of Caspase‐3, Bcl‐2 and EMT‐related proteins were further detected (Figure 7J,K and Figure S5H,I). Furthermore, we found that FOXP2 knockdown reversed the increase in GFP/mRFP‐LC3 dots caused by transfection with miR‐300 inhibitors in GC cells (Figure 7H,I and Figure S5F,G). Additionally, knockdown of miR‐300 raised the rate of LC3 II/I and reduced the level of P62, which could be recovered by cotransfection with FOXP2 siRNAs (Figure 7J,K and Figure S5H,I). Combined with the above results, we proved that circST3GAL6 markedly regulates FOXP2 expression and promotes autophagy by sponging miR‐300.

**FIGURE 7:** Knockdown of Forkhead box P2 (FOXP2) reverses the effect of miR‐300 inhibitors on gastric cancer (GC) cells. (A,B) Knockdown of FOXP2 could restore the effect of miR‐300 inhibitors on cell proliferation in BGC‐823 and SGC‐7901 cells by colony formation assays. (C,D) Knockdown of FOXP2 could restore the effect of miR‐300 inhibitors on cell proliferation in BGC‐823 and SGC‐7901 cells by 5‐ethynyl‐2′‐deoxyuridine (EdU) assays, scale bar = 100μm. (E) The promotion of cell apoptosis by miR‐300 inhibitors was restored by knockdown of FOXP2 in BGC‐823 and SGC‐7901 cells. (F,G) The inhibition of cell migration and invasion by miR‐300 inhibitors was restored by knockdown of FOXP2 in BGC‐823 and SGC‐7901 cells. (H,I) The effect of miR‐300 inhibitors on autophagy can be recovered by knockdown of FOXP2 in BGC‐823 and SGC‐7901 cells, scale bar = 20μm. (J,K) Expression levels of apoptotic, epithelial‐mesenchymal transition (EMT) and autophagy proteins were examined by western blotting in BGC‐823 and SGC‐7901 cells. (*p < .05, **p < .01, ***p < .001. Data are expressed as the means ± SDs)

RETRACTED

### 3.9 FOXP2 transcriptionally inhibits MET and regulates autophagy

We proved that circST3GAL6 promoted autophagy via the miR‐300/FOXP2 axis, but the downstream mechanism of FOXP2 remains to be explored. FOXP2 was reported to be a transcription factor that could bind to the MET promoter and inhibits its expression.^18^ The negative correlation between FOXP2 and MET was confirmed from the TCGA database (Figure S6A). As a receptor tyrosine kinase, MET mediates signal transduction from the extracellular matrix to the cytoplasm and impacts several biological behaviours, such as proliferation, metastasis, and drug resistance. On the basis of the above results, we tried to investigate whether FOXP2 regulated autophagy through MET. Next, we searched the possible binding sites with FOXP2 on the promoter of MET 0–2000 bp upstream using JASPAR (Figure 8A). Two possible binding sites were confirmed according to the binding score (Figure 8A). We constructed three PGL3 luciferase reporter gene vectors of FOXP2 promoter regions that covered the potential binding sites (Figure 8A). FOXP2 overexpression significantly reduced the luciferase activity of P1 rather than P3, indicating that the 1000 region was the junction site between FOXP2 and MET promoter (Figure 8B). Furthermore, the binding sites between FOXP2 and MET promoters were determined by the ChIP assay. The amplification of the pulled‐down DNA with Primer 2 was significantly stronger than that with Primer 3, which was demonstrated via qRT‐PCR (Figure 8C,D and Figure S6B). These results showed that FOXP2 directly bonded to binding site A on the promoter of MET. MET activates downstream signalling pathways, including the PI3K‐Akt‐mTOR pathway, a classical pathway regulating autophagy.^32^, ^33^ The downstream signalling pathway of FOXP2 was detected by western blotting assay. Knockdown of FOXP2 upregulated the expression levels of MET, phospho‐AKT (T308, S473) and phospho‐mTOR (S2448) and these effects were reversed by MET silencing (Figure 8E and Figure S6D,E). Knockdown of FOXP2 could downregulate the rate of LC3 II/I while the expression of P62 was upregulated, which could be restored by downregulated MET (Figure 8E and Figure S6D,E). These results were also confirmed by GFP/mRFP‐LC3 dot analysis and TEM (Figure 8F and Figure S6C). Furthermore, we investigated whether GC cell proliferation and migration affected by circST3GAL6 through FOXP2 were regulated by autophagy. Note that, 3‐MA (3‐methyladenine), an autophagy inhibitor was applied to further study. FOXP2 overexpression promoted autophagy, which could be suppressed by 3‐MA through GFP/mRFP‐LC3 dots, TEM and western blotting (Figure 8H–J and Figure S7A,B,G). Subsequently, FOXP2 overexpression could inhibit cell proliferation and metastasis, which could be restored by 3‐MA (Figure 8K–N and Figure S7C–F). Thus, we demonstrated that circST3GAL6 regulated the AKT/mTOR pathway through FOXP2 transcriptional inhibition of MET to affect autophagy, thus regulating the proliferation and metastasis of GC (Figure 9A).

RETRACTED

**FIGURE 8:** Forkhead box P2 (FOXP2) transcriptionally inhibits MET and regulates autophagy through AKT/mTOR axis which regulates the malignant progression of gastric cancer (GC) cells. (A) Schematic diagram showed three luciferase reporters cover different DNA sequences of MET promoter region. (B) Luciferase reporter assay analysis of three MET promoter luciferase reporters in BGC‐823 cells transfected with FOXP2 or pcDNA. (C) Schematic diagram showed three primers for ChIP assay. (D) Quantitative real‐time polymerase chain reaction (qRT‐PCR) was performed in BGC‐823 cell after pulling down FOXP2 using three pairs of primers to investigate the potential FOXP2 binding sites in MET promoter region. (E) Expression levels of FOXP2, MET/AKT/mTOR and autophagy proteins were examined by western blotting. (F,G) The effect of overexpression of circST3GAL6 on autophagy can be recovered by knockdown of FOXP2 via confocal microscopy (scale bar = 20μm) and transmission electron microscopy scale bar = 1μm in BGC‐823 cell. (H,I) The effect of overexpression of FOXP2 on autophagy can be recovered by 3‐methyladenine (3‐MA; 5 nM, 24 h) via confocal microscopy (scale bar = 20μm) and transmission electron microscopy (scale bar = 1μm) in BGC‐823 cell. (J) Expression levels of autophagy‐related proteins were examined by western blotting in BGC‐823 cell. (K–M) 3‐MA (5 nM, 24 h) could restore the effect of FOXP2 overexpression on cell proliferation in BGC‐823 cell by CCK8, colony formation and 5‐ethynyl‐2′‐deoxyuridine (EdU) assays. (N) 3‐MA (5 nM, 24 h) could restore the effect of FOXP2 overexpression on cell migration and invasion in BGC‐823 cell transwell assays. (*p < .05, **p < .01, ***p < .001. Data are expressed as the means ± SDs)

**FIGURE 9:** The mechanism diagram of circST3GAL6/miR‐300/FOXP2 axis

RETRACTED

## 4 DISCUSSION

Gastric cancer ranks fifth in incidence among all cancers worldwide, and its incidence is particularly high in East Asia, including China.^1^, ^2^ New targets are warranted for GC treatment. We performed the next‐generation sequencing assay to study the differential expression profile of circRNAs in gastric cancer. After screening the sequencing results, circST3GAL6 was selected because of its highest foldchange, which may play a significant role in GC. This is the first report showing the circular RNA ST3GAL6 can inhibit the malignant progression of gastric cancer. According to previous studies, linear ST3GAL6 participated in the development of multiple tumours, such as urinary bladder cancer, CRC and multiple myeloma,^34^, ^35^, ^36^ suggesting a potential connection between the two forms. Furthermore, circST3GAL6 expression was correlated with clinical stage and tumour size, which was expected to be one of the biomarkers for detecting gastric cancer.

CircRNAs affect cancer progression by sponging miRNA or RNA‐binding proteins (RBPs),^37^ they can even be translated into proteins.^38^ We proved that circST3GAL6 could sponge miR‐300, forming a natural competitive endogenous RNA network. Our results confirmed that in both GC cell lines, only miR‐300 could be pulled down via the circST3GAL6 probe. Several reports demonstrated that circRNAs could impact RBPs and that some RBPs could even affect the expression of circRNAs in turn.^39^ The mutant plasmid that blocked the connection between circST3GAL6 and miR‐300 confirmed that the suppressive role of circST3GAL6 was miR‐300 dependent. However, circST3GAL6 MUT did not restore the effect of circST3GAL6 totally. We tried to predict whether some RBPs could bind to circST3GAL6 via RBPmap (http://rbpmap.technion.ac.il/), and the results showed that KHDRBS1 might have a connection with circST3GAL6. Although KHDRBS1 promoted pre‐mRNA circularization, we found that KHDRBS1 could not affect the expression of circST3GAL6 when it was knocked down. There may be some potential RBPs still to be discovered.

The FOXP family is considered to be a group of transcription factors,^14^ and FOXP2 was predicted and identified as the target gene of miR‐300. Because FOXP2 played a vital role in regulating gene transcription, we predicted the potential binding sites of the MET promoter via JASPAR.^18^ The transcription of MET via FOXP2 was verified by the luciferase assay and ChIP assay. MET is a kind of receptor tyrosine kinases. The MET receptor binds to its ligand, hepatocyte growth factor, to induce the dimerization of MET, entering an active state, where it phosphorylates its substrate and activates downstream pathways, including the MAPK/ERK and PI3K‐Akt‐mTOR pathways.^40^, ^41^ Since circST3GAL6 regulated autophagy in our previous experiments and circST3GAL6 could affect MET by binding FOXP2 via miR‐300, we further verified whether circST3GAL6 could affect autophagy via the FOXP2/MET axis. CircST3GAL6 further regulated autophagy by affecting mTOR phosphorylation through FOXP2‐mediated MET transcriptional inhibition. Furthermore, we found that GC cell proliferation and migration were altered after applying the autophagy inhibitor 3‐MA. Although autophagy was reported to regulate cell proliferation, migration and apoptosis,^42^, ^43^, ^44^, ^45^ the specific mechanism needs to be explored and confirmed in vivo.

RETRACTED

## 5 CONCLUSION

CircST3GAL6 was significantly reduced in GC cells and tissues. Overexpression of circST3GAL6 suppressed the malignant progression of GC through autophagy, which was regulated by FOXP2/MET/mTOR axis. In conclusion, the above results proved that circST3GAL6 might become a potential therapeutic target for GC in the future.

## CONFLICT OF INTEREST

The authors declare that they have no conflict of interest.

## Supporting information



Supporting Information

Supporting Information

Supporting Information

Supporting Information

Supporting Information

Supporting Information

Supporting Information

Supporting Information

Supporting Information
